# A Study on the Relationship between Mental Resilience, Work-Family Conflict, and Anxiety of Nurses in Shandong, China

This article has been retracted.

**DOI:** 10.1155/2022/4308618

**Published:** 2022-03-02

**Authors:** Qin Qi, Xiaoyun Yan, Meng Gao, Xia Wu, Shuhong Zhang, Ronnell D. Dela Rosa, Yan Zhang, Yuzhen Xu

**Affiliations:** ^1^Taian City Central Hospital, Taian, Shandong 271000, China; ^2^Taian City First People's Hospital, Shandong 271000, China; ^3^Bataan Peninsula State University, College of Nursing and Midwifery, City of Balanga, 2100, Bataan, Philippines; ^4^Philippine Women's University, School of Nursing, Manila 1004, Philippines; ^5^The Second Affiliated Hospital of Shandong First Medical University, Taian, Shandong 271000, China

## Abstract

Based on Freud's personality theory, 839 nurses from 5 public hospitals in Shandong Province were selected by the convenience sampling method. A cross-sectional survey was conducted to investigate the correlation among resilience, work-family conflict (WFC), and anxiety (SAS). The purpose of this study was to explore the relationship among resilience, WFC, and SAS of these nurses and to provide evidence with reducing WFC and SAS for the nurses. The results showed that the total score of resilience, WFC, and SAS was 58.00 ± 18.27, 53.46 ± 13.29, and 49.98 ± 14.73, respectively. There was 47.68% of the nurses that had anxiety, and 10.97% of the nurses had severe anxiety. There were significant differences in the score of SAS among the length of service, self-perceived health status, confidence in nursing professional development, WFC, and resilience (*P* < 0.05). This study draws the following conclusions: the proportion of anxiety is high, and the level of resilience is lower than the domestic norm. Length of service, self-perceived health status, confidence in nursing professional development, WFC, and resilience were the important influencing factors of anxiety. It is suggested that hospital managers should pay attention to the mental health of nurses, take active intervention measures according to the influencing factors of SAS, improve nurses' psychological resilience, reduce WFC and anxiety, improve nurses' mental health and well-being, and ensure nursing safety.

## 1. Introduction

With the development of science and technology, the people have an increasing demand for health. Nurses would be required with more professional knowledge and skills. Nurses often encounter stress and work-related conflicts, such as busy work, taking care of paining and dying patients, extending work hours, doing technical difficulty, and rescuing critically ill patients [1, 2]. It can easily lead to psychological problems of nurses [1, 2]. SAS is one of the most common psychological disorders [3]. The study showed that 32-43% of nurses in HK [4], 20% of midwives in Australian [5], and 44-66% of nurses in Brazilian [6] have mental disorders. This mental health problem has adverse effects on occupational performance and well-being and may lead to a decline in the quality of patient care and safety problems [1, 7].

Working family problem is an important factor in the field of occupational health psychology [8]. Nurses are mostly women and play the role caregiver in the families. Many nurses have more than 2 kids with the policy of China's two-child implemented from 2014, and the task of taking care of the family is more heavy. Due to busy work and emotional fatigue, nurses do not have much energy to take care of their families, resulting in WFC [9, 10]. WFC will not only affect the career development of nurses [11], but also lead to nurse mental health problems [12].

Psychological resilience refers to the good adaptation process [13] of individuals in the face of negative events such as adversity, trauma, tragedy, threat, or other major stress, which is an important psychological variable affecting the ability of self-regulation. Nurses with strong psychological resilience can actively face and quickly adjust themselves to stress sources and negative events, achieve a new balance, and reduce the impact on mental health [14–16].

At present, there is less research on the psychological resilience and WFC and SAS association effect of nurses. This study is aimed at understanding the status of psychological resilience, WFC, and SAS mood of nurses in Shandong of China, and to analyze the important influencing factors leading to the nurse SAS. It provides an empirical basis for hospital managers to take intervention measures against the influencing factors to improve the mental health and well-being of nurses.

Freud's theory stated that personality is composed of id, ego, and superego. The components of id are the basic needs of human beings. The impulse of ego to ID and the control of superego have the function of buffering and regulating. Superego is formed by individuals accepting social and cultural moral norms. The three levels of personality structure interweave with each other to form an organic whole, thus ensuring the normal development of personality. If the three levels are out of balance, it will lead to psychological disorders [17]. If nurses often work night shift, it will affect their sleep and id. Nurses on night shift cannot take care of family and children, which will affect superego. The continuous occurrence of conflicts will lead to anxiety emotions among nurses.

## 2. Methods

### 2.1. Study Population

This study was a descriptive cross-sectional research design. In this study, the convenience sampling method was used to select nurses from public hospitals in Shandong Province. The inclusion standard was as follows: (1) had nurse qualification certificate and working for more than 1 year and (2) voluntary participation in this study. The exclusion criteria were as follows: having the qualification certificate but not working in the hospital. Using the G-Power 3.1.9 software program (Heinrich Heine University, Dusseldorf, Germany), according to the multiple regression analysis, the significance level was 0.05, the median validity was 0.15, and the power was 95.0%; there were 21 predictors (18 demographic characteristics, resilience, WFC, SAS). The estimated sample size is 472.

In this study, quality control was adopted to ensure the reliability of the results. First, 60 nurses from a hospital were randomly selected for presurvey according to the predesigned questionnaire to verify the feasibility of the study and rectify the existing problems. From May to June 2021, the investigators organized the training in each hospital as a third party, with the support of the managers of the sampled hospitals, and questionnaire survey was conducted among nurses with voluntary participation. In order to reduce manual input errors, an app was designed about the questionnaire to fill in the questionnaire by their mobile phones. A total of 839 questionnaires were issued, and all the questionnaires were valid and no logical errors.

The ethics committee of Taian Central Hospital approved the study (approval number No. 2021-5-14). The investigator explained the purpose and procedure of the study in detail to all nurses participating in the survey and clarified the voluntary nature and confidentiality of the study. Nurses participated in the study with informed consent.

### 2.2. Psychological Resilience

Resilience scale was drawn up by Connor and Davidson [18] and translated and revised by Xin and Zhang [19]. It has 25 items and three dimensions of resilience, strength, and optimism. The test-retest reliability of the scale was 0.87, and Cronbach's *α* was 0.89, which was widely used in clinic [20, 21]. Likert 5-level scoring method was used in the scale. The items from “never” to “almost always” were 0-4 points in turn. The sum of the scores was the total score. The higher the total score was, the better the resilience was.

### 2.3. Work-Family Conflict

Work-family conflict (WFC) was developed by Carlson [22] and revised by Zhang [23], with 18 items and 3 dimensions. They are time-based conflict, pressure-based conflict, and behavior-based conflict. Cronbach's *α* is 0.859, and Cronbach's *α* is 0.789~ 0.878 of each dimension. The scale adopts a Likert 5 score of 18~ 90. The higher the score, the stronger the conflict.

### 2.4. SAS

Anxiety symptoms were measured using the Zung SAS Self-Evaluation Scale [24]. This Chinese version chose SAS for study [25]. SAS has 20 items with a level Likert 4 scoring method. Cronbach's *α* is 0.71. The score of SAS was divided into none (25-49), mild (50-59), moderate (60-69), and severe (70-100). The higher the score, the higher the anxiety [26].

### 2.5. Statistical Analysis

The data were analyzed by SPSS 20.0 (IBM Corporation, Armonk, NY). The total psychological resilience score, work-family conflict total score, and SAS total score for normality test showed a normal distribution. Measurement data is expressed by mean standard difference, psychological resilience, work-family conflict, and SAS relationship using Pearson correlation analysis, and multifactor analysis adoptslinear regression analysis < 0.05that has statistical significance.

## 3. Results

### 3.1. General Data and SAS Single Factor Analysis of the Research Subjects

The average age was 31.88 ± 6.49 years, and the average length of service was 9.92 ± 6.98 years of 839 subjects.  Table 1 presents general data of these nurses, such as the means and standard deviations.

The results of SAS single factor analysis (Table 1) showed that there was significant difference in SAS score among nurses (*P* < 0.05), such as the department, length of service, education background, number of conflicts with caregivers, time spent on the way to work, self-perceived health status, consistency between income and work, average number of night shifts per month, harmony with colleagues, satisfaction with working environment, confidence in nursing career development, and reasons for choosing a nurse's career. Nurses in intensive care unit, working for 6-10 years and have bachelor's degree, had high anxiety. The more night shift, the more anxiety. The nurses who felt that they were in poor health and had no choice but to choose nursing specialty showed moderate anxiety. The nurses who thought that the income was not consistent with the payment and had no confidence in the development of nursing profession showed mild anxiety. Nurses who did not get along well with their colleagues and were extremely dissatisfied with the working environment showed severe anxiety.

According to SAS score: no (25-49), mild (50-59), moderate degree (60-69), and severe (70-100), the SAS ratio is shown in Table 2.

Table 2 shows that 47.68% of the subjects had anxiety and 10.97% had severe anxiety.

### 3.2. The Score of SAS, the Psychological Resilience, and WFC of the Nurses

The total SAS score, psychological resilience, and WFC score of nurses in the Shandong region are shown in Table 3.

### 3.3. Correlational Analysis of SAS, WFC, and Psychological Resilience of the Nurses

The analysis results of SAS, WFC, and psychological resilience of the nurses are shown in Table 4.

### 3.4. Multiple Regression Analysis of SAS Influencing Factors

The total score of SAS was taken as the dependent variable, and the variables influencing the positive of SAS single factor analysis (such as department, length of service, education background, WFC, and resilience) were taken as the independent variables. The results of multiple linear regression analysis were shown in Table 5.

The main factors influencing SAS scores were length of service, self-consciousness and health status, confidence in nursing professional development, WFC, and psychological resilience. The difference of SAS scores was significant (*P* < 0.05).

## 4. Discussion

Shandong is located in the north of China, which is a medium developed area. The treatment and management of nurses are similar to that of most regions in China, which has a certain regional representation. The results showed that 47.68% of nurses had SAS emotion, and 10.97% had severe SAS. Length of service, perceived health status, confidence in the development prospects of nursing profession, WFC, and resilience were the important influencing factors of nurses' anxiety.

Nurses who have worked for 6-10 years have mastered certain knowledge and skills and have more thoughts on the sense of work value and career development direction. At the same time, it is in the peak period of love, marriage, and childbearing. Faced with many choices and conflicts, SAS is easy to appear.

The SAS score of nurses with poor health was 65.34 ± 15.89, showing moderate anxiety. This may be related to the working environment of nurses. Nurses have a large workload and high risk, especially ICU nurses, who take care of critically ill patients who need rescue or dying at any time. It is easy to cause physical loss and psychological fatigue of nurses and increase job burnout and anxiety [27].

Nurses who had no confidence in nursing professional development showed moderate anxiety. According to Freud's personality theory, nurses have no confidence in their work and cannot feel the sense of professional value and achievement, which will cause them to lose their motivation and anxiety.

This study shows that WFC is an important influencing factor of nurses' anxiety, which is consistent with the related studies that WFC can lead to physical and psychological problems [28, 29]. The time-based conflict and stress-based conflict of nurses in Shandong were higher than 3 points. The conflict index based on time is the highest. This has something to do with the irregular life of nurses, working night shift, and even not being able to get off work on time when encountering emergency patients. The nurses who worked more than 11 night shifts per month had obvious anxiety. Sleep is an important factor for nurses to recover from fatigue and psychological stress [30]. WFC was positively correlated with sleep deprivation [31]. The more time nurses spend on work and on the road, the less time they spend on taking care of their families. In the work to pay too much energy, in the return to the family, due to fatigue cannot take good care of the family. High level of WFC may affect job performance and lead to psychological depression of nurses [32].

The total score of resilience was 58.00 ± 18.27, which was lower than the domestic norm of 65.4 ± 13.9 [33]. The optimistic index is the lowest. Resilience is a dynamic process of psychological adjustment in the face of negative events. The stronger the resilience, the faster the adjustment speed to adapt to the new environment, and the smaller the impact on mental health. The meaning of process based resilience is that “time” factor needs to be considered [15]. The working environment of the hospital leads to long-term pressure of nurses. Long-term chronic stimulation will lead to the decline of psychological adjustment ability, and it is difficult for nurses to maintain optimistic psychology due to job burnout [34].

This study provides an empirical basis for hospital managers to take intervention measures to reduce nurses' SAS. Managers should pay attention to the mental health of nurses, especially the nurses who have worked in the intensive care unit for a long time, the nurses who have worked for 6-10 years, the nurses who have been on duty for many times at night, and the nurses who feel unhealthy. We can adjust the position appropriately, carry out career development planning and professional value education for nurses, and guide them to have full confidence in the nursing profession. The nurses with anxiety were given psychological counseling in time. For nurses who work far away from home, convenient transportation can be provided, such as setting up shuttle bus and improving the working environment. The nurses were trained in the knowledge of communication and resilience, and their communication ability and emergency response ability were strengthened. Regularly carry out recreational activities to improve their psychological state and harmonize the relationship between colleagues and family members. Reducing the WFC of nurses and improve the resilience can reduce the anxiety of nurses. Nurses are the direct caregivers of patients, and their mental health is helpful to provide patients with high quality and safe nursing service.

The study also has some limitations. First of all, this study is a cross-sectional study, the data source is the participants' self-administered questionnaire, there are subjective factors, and the results of the data may be questioned. Qualitative study and longitudinal cohort study will be added in the future study. Secondly, this study uses the convenient sampling method to select participants instead of random sampling, which may lead to bias of results. Future studies can retest the validity of the results in additional samples. Finally, most of the subjects in this study are women, which may lead to gender bias. Future research can increase the survey of male nurses.

## 5. Conclusion

This study conducted a cross-sectional questionnaire survey among nurses in 5 hospitals in Shandong Province of China and analyzed the correlation between resilience, WFC, and SAS. The proportion of SAS is high. Length of service, perceived health status, confidence in nursing professional development, WFC, and resilience were the important influencing factors of SAS emotion. WFC was positively correlated with SAS and negatively correlated with resilience. SAS was positively correlated with resilience.

## Figures and Tables

**Table 1:** Analysis of survey object general data and SAS point single factor analysis.

The project	Number (*n*, %)	Points $\left(\bar{x}\pm s\right)$	*t*/*F*	*P*
The department			4.331	0.013
Monitoring room	314 (37.43)	51.84 ± 16.08		
Internal medicine	295 (35.16)	48.45 ± 13.44		
Surgery	230 (27.41)	49.38 ± 14.16		
Gender			1.414	0.501
Male	48 (5.72)	52.89 ± 14.01		
Female	791 (94.28)	49.8 ± 14.76		
Age			2.422	0.065
20~ 30	376 (44.82)	49.03 ± 14.86		
31~ 40	380 (45.29)	51.27 ± 14.69		
41~ 50	76 (9.06)	48.96 ± 13.70		
51 up	7 (0.83)	41.43 ± 15.84		
Length of service			8.297	≤0.001
1 ~ 5	227 (27.06)	46.33 ± 13.98		
6 ~ 10	304 (36.23)	52.08 ± 15.11		
11~ 20	227 (27.06)	51.54 ± 14.48		
21 up	81 (9.65)	47.9 ± 14.03		
Education			5.379	0.005
Junior college	100 (11.92)	45.83 ± 14.69		
Bachelor degree	729 (86.89)	50.62 ± 14.68		
Master's degree and above	10 (1.19)	44.63 ± 11.04		
Marriage status			2.216	0.110
Married	638 (76.04)	50.55 ± 14.57		
Divorced and widowed	6 (0.72)	44.79 ± 15.62		
Unmarried	195 (23.24)	48.24 ± 15.13		
Number of children			2.424	0.089
No children	259 (30.87)	48.36 ± 15.03		
1 child	358 (42.67)	50.42 ± 14.93		
More than 2 children	222 (26.46)	51.14 ± 13.92		
Children caregivers			1.401	0.241
Not so involved	274 (32.66)	48.58 ± 15.33		
Parents	381 (45.41)	50.95 ± 14.27		
Myself or husband	178 (21.22)	49.98 ± 14.86		
Babanny or others	6 (0.72)	51.67 ± 6.55		
Frequency of a conflict with the caregiver			21.668	≤0.001
Often	111 (13.23)	59.47 ± 16.09		
Sometimes	256 (30.51)	50.26 ± 12.35		
Very few	225 (26.82)	48.55 ± 14.22		
Never	247 (29.44)	46.71 ± 15.09		
Willingness to have three children			0.707	0.494
Yes	17 (2.03)	53.6 ± 14.61		
No	706 (84.15)	50.02 ± 14.67		
Unsure	116 (13.83)	49.14 ± 15.13		
Number of night shift per month			4.818	0.008
No night shift	158 (18.83)	47.77 ± 13.55		
1 ~ and 10	575 (68.53)	49.93 ± 14.83		
More than 11 people	106 (12.63)	53.48 ± 15.31		
Take time on the way to work every day			7.294	0.001
Within 30 minutes	618 (73.66)	48.82 ± 14.06		
30~ 60 minutes	197 (23.48)	53.15 ± 15.96		
More than 60 minutes	24 (2.86)	53.59 ± 17.13		
Self-perceived health status			114.283	≤0.001
Health	284 (33.85)	42.71 ± 12.14		
General rule	456 (54.35)	51.17 ± 12.95		
Difference	99 (11.8)	65.34 ± 15.89		
Is the income consistent with the work			7.243	0.005
Conformity	197 (23.48)	43.52 ± 12.41		
Not consistent	642 (76.52)	51.95 ± 14.82		
Confidence in career prospects			58.486	≤0.001
Full confidence	594 (70.8)	46.73 ± 13.18		
Not concerned	54 (6.44)	54.65 ± 14.71		
No confidence	190 (22.65)	58.82 ± 15.40		
Relationship with colleagues			25.974	≤0.001
Harmony	685 (81.64)	48.51 ± 14.08		
General rule	149 (17.76)	55.74 ± 15.45		
Not so harmonious	5 (0.60)	79.00 ± 5.69		
Evaluation of working environment			5.319	≤0.001
Very satisfied	154 (18.36)	42.50 ± 12.33		
More satisfied	287 (34.21)	46.64 ± 12.42		
General rule	302 (36)	53.03 ± 13.82		
Less satisfied	59 (7.03)	57.78 ± 14.80		
Very dissatisfied	37 (4.41)	69.59 ± 18.08		
Purpose of occupation			16.662	≤0.001
To make a living	524 (62.46)	52.49 ± 14.95		
Self-value realization	252 (30.04)	44.40 ± 12.58		
Forced to do	11 (1.31)	64.20 ± 15.93		
Unsure	44 (5.24)	48.84 ± 14.15		
Affected by others	8 (0.95)	47.66 ± 9.17		

**Table 2:** Degree of SAS (n, %).

The project	No SAS	SAS mood		
		Mild	Moderate degree	Severe
Number of people	439	209	99	92
The portion	52.32	24.91	11.80	10.97

**Table 3:** Score of SAS, WFC, and resilience of nurses $\left(\bar{x}\pm s\right)$.

The project	Number of items	Total score	Item score	Index value (%)	Order
SAS	20	49.98 ± 14.73	2.00 ± 0.88	62.48	—
WFC	18	53.46 ± 13.29	2.97 ± 0.74	59.40	—
Time-based conflicts	6	18.42 ± 4.89	3.07 ± 0.81	61.40	1
Pressure-based conflict	6	18.04 ± 4.86	3.01 ± 0.81	60.13	2
Behavioral-based conflicts	6	17.00 ± 5.23	2.83 ± 0.87	56.67	3
WFC to the families	9	29.26 ± 7.62	3.25 ± 0.85	65.02	1
WFC to the work	9	24.21 ± 7.07	2.69 ± 0.79	53.80	2
Psychological resilience	25	58.00 ± 18.27	2.32 ± 0.73	46.39	—
Attitude	13	29.20 ± 10.05	2.25 ± 0.77	44.92	2
Strength	8	19.81 ± 6.00	2.48 ± 0.75	49.53	1
Optimism	4	8.98 ± 3.17	2.24 ± 0.79	44.92	3

Note: index value = actual score/theoretical maximum score × 100%.

**Table 4:** The correlational analysis results of SAS, WFC, and psychological resilience.

Variable	1	2	3	4	5	6	7	8
1. SAS	1							
2. Time conflicts	0.468^∗∗^	1						
3. Pressure conflict	0.542^∗∗^	0.748^∗∗^	1					
4. Behavioral conflicts	0.507^∗∗^	0.593^∗∗^	0.702^∗∗^	1				
5. WFC	0.570^∗∗^	0.875^∗∗^	0.918^∗∗^	0.869^∗∗^	1			
6.Fortitude	-0.323^∗∗^	-0.217^∗∗^	-0.315^∗∗^	-0.290^∗∗^	-0.309^∗∗^	1		
7. Strength	-0.345^∗∗^	-0.236^∗∗^	-0.331^∗∗^	-0.331^∗∗^	-0.338^∗∗^	0.896^∗∗^	1	
8. Optimistic	-0.292^∗∗^	-0.202^∗∗^	-0.287^∗∗^	-0.274^∗∗^	-0.287^∗∗^	0.759^∗∗^	0.792^∗∗^	1
9. Resilience	-0.342^∗∗^	-0.232^∗∗^	-0.332^∗∗^	-0.316^∗∗^	-0.331^∗∗^	0.976^∗∗^	0.959^∗∗^	0.851^∗∗^

Note: ^∗∗^significant correlation at 0.01 level (bilateral).

**Table 5:** The results of multiple regression analysis of SAS (*n* = 839).

Variable	*B*	Standard error	Standard coefficient	*t*	*P*
(Constant)	14.497	5.201		2.787	0.005
Length of service	1.050	0.479	0.067	2.192	0.029
Health state	5.555	0.676	0.241	8.219	≤0.001
Confidence in career prospects	1.795	0.535	0.102	3.358	0.001
WFC	0.450	0.033	0.406	13.651	≤0.001
Resilience	-0.065	0.024	-0.080	-2.738	0.006

Note: *R* = 0.673, *R*^2^ = 0.453, adjust *R*^2^ = 0.443, *F* = 48.680, *P* < .05.

## Data Availability

The data utilized which corroborated this study's conclusions are accessible once requested from the corresponding author.
